The article "Reform and Analysis of the Division of Legal Responsibility between Enterprises and Third-Party Governance under Environmental Pollution" was published in 2022. Journal: J Environ Public Health.

# Reform and Analysis of the Division of Legal Responsibility between Enterprises and Third-Party Governance under Environmental Pollution

**DOI:** 10.1155/2022/5168699

**Published:** 2022-06-23

**Authors:** Yijun Wu

**Affiliations:** School of Law, Anhui University, Hefei, Anhui 230000, China

## Abstract

This paper aims to deeply analyze the relevant concepts of the third-party responsibility for environmental pollution control of enterprises and further clarify the legal responsibility and responsibility distribution of the third-party environmental pollution control. Through the analysis of enterprise environmental pollution sample data, this paper finds that the judicial application of enterprise environmental pollution crime in China mainly includes the number of cases increases year by year and the subjects of enterprise environmental pollution crime are relatively concentrated. The results show that the joint crime accounts for about 40%, and unit crime cases account for about 10%, while the amount of fines for natural persons in the existing laws is mostly less than 50,000 yuan, which is relatively low. Finally, it is concluded that the criminal punishment of enterprise environmental pollution is relatively light, especially in the accountability of the criminal subject. Therefore, this paper focuses on the division of legal liability from three aspects: civil liability, administrative liability, and criminal liability.

## 1. Introduction

In recent years, with the intensification of environmental problems, the third-party governance of environmental pollution has received extensive attention. Based on the traditional “who pollutes, who governs” model and principle, it is difficult for the subject of environmental pollution to achieve efficient environmental governance due to the lack of pollution control ability and technical defects [1]. Although the government undertakes the main responsibility of environmental governance in the public sphere in the process of environmental governance, it is unable to make scientific decisions due to the lack of professional pollution control talents and scientific management means. The transformation of the third-party governance mode of enterprise environmental pollution is directly related to the promotion of national policies. However, due to the fact that the national case responsibility in this regard has not been clearly clarified, the distribution of responsibility for the third-party governance is not clear enough, especially the internal responsibility defects have caused some obstacles to the third-party governance. Therefore, aiming at the existing problems, this paper focuses on the definition of the third-party governance responsibility in enterprise environmental pollution from the legal level. See Figure 1.

The article "Reform and Analysis of the Division of Legal Responsibility between Enterprises and Third-Party Governance under Environmental Pollution" was published in 2022. Journal: J Environ Public Health.

## 2. Literature Review

In terms of the legal background of environmental governance abroad, some developed countries will not only stipulate the responsibilities and obligations of governments, enterprises, social organizations, and citizens at all levels by issuing relevant laws but also encourage enterprises to entrust the pollution control work to licensed professional environmental service companies, which provides a guarantee for the marketization of environmental protection industry. In practice, according to relevant laws and regulations, a strict review and licensing system for pollution control enterprises is implemented, and different pollutant treatment practitioners need to go through different levels of qualification review and certification processes. In addition, the law focuses on the discharger's responsibility and extended producer's responsibility. The discharger is responsible for the discharged industrial waste, and the producer is responsible for the pollution generated in the whole life cycle of the product. If the regulations are violated, the local governor can exercise the power of supervision and inspection to punish them. In the third-party governance model of enterprise environmental pollution, how to allocate legal responsibility has become the focus of theoretical and practical circles [2, 3]. At present, there are mainly the following four views:

First, it advocates that the responsibility should be borne by the pollutant discharge enterprise, that is, if the discharge still fails to meet the standard after being treated by a third party, the pollutant discharge enterprise should bear the corresponding legal responsibility independently, and the third party should not bear the responsibility.

Second, it advocates that the third party should bear the responsibility, that is, the environmental service company should bear the corresponding legal responsibility if the discharge still fails to meet the standard after being treated by the third party.

Third, it advocates to assume responsibility according to the agreement, that is, the responsibility should be defined according to the specific content of the contract signed between the pollutant discharge enterprise and the third party, the mode of cooperation, and the degree of fault in the performance of the contract. In short, those who breach the contract will bear the responsibility; for example, scholars have proposed that if the third party strictly performs the contract, but the pollutant discharge enterprise discharges excessive pollutants or commits other acts in violation of the terms of the contract, the pollutant discharge enterprise should bear the responsibility.

The article "Reform and Analysis of the Division of Legal Responsibility between Enterprises and Third-Party Governance under Environmental Pollution" was published in 2022. Journal: J Environ Public Health.

Fourth, it advocates that the responsibilities should be determined according to the comprehensive situation. Some scholars propose that the modes of “entrusted governance service” and “entrusted operation service” should be distinguished to determine the primary and secondary responsibilities. Some scholars divide the third-party governance model of “enterprise cooperation” into independent and embedded types and determine the commitment of environmental tort liability respectively according to the fault of sewage enterprises and third-party governance [4, 5].

## 3. Legislative Evolution of Environmental Pollution Crime

Since the eighth punishment, the crime of polluting the environment has officially replaced the previous crime, opening a new era of environmental crime control. The crime of polluting the environment, which has been revised since the Eleventh Amendment to the criminal law, is no longer a minor crime in the early days of its establishment, but a felony [6]. At the same time of the crime of polluting the environment, if a heavier crime is committed, such as the crime of putting dangerous substances, the crime can be sentenced to death at most, which enhances the deterrence of the crime of polluting the environment. Therefore, the newly revised crime of polluting the environment improves the current situation of low sentencing of the crime of polluting the environment and increases the punishment of the crime of polluting the environment. See Tables 1 and 2.

## 4. Sample Analysis of Judicial Application Cases of Environmental Pollution Crime

### 4.1. Sample

Based on this explanation, relevant departments continued to maintain a high pressure on environmental pollution crimes, resolutely punished corresponding criminal activities, and achieved good social results. The author searched the two key words of criminal cases and environmental pollution crime on the judgment document network and found a total of 16,140 documents, covering 31 provinces and cities and a construction corps (see Table 3).

It can be seen from the above table that among the 16,140 documents retrieved on the judgment document network, 12,698 were first instance by the grassroots courts and 55 were first instance by the intermediate courts. Generally speaking, the cases involving the crime of environmental pollution are of great social harm and deserve attention; for example, the Tengger Desert pollution case eventually caused ecological losses, and the contaminated soil area was about 120,000 square meters, about 180 mu. Finally, the eight enterprises involved shared the repair cost of 560 million yuan. Although there are few such cases, the impact is unprecedented and needs our attention [7–9].

The article "Reform and Analysis of the Division of Legal Responsibility between Enterprises and Third-Party Governance under Environmental Pollution" was published in 2022. Journal: J Environ Public Health.

It can be seen from Figure 2 that the number of criminal cases of environmental pollution crime has increased significantly since the implementation of the “13 interpretation.” It was not until 2017 that the number of environmental pollution crime cases closed reached a breakthrough from single digits to ten digits, with 39 cases. In 2018, the number of environmental pollution crime cases closed reached 944, showing an explosive growth. Until the end of 2020, the number of closed cases began to show a downward trend [10]. By the end of 2020, the number of closed criminal cases of environmental pollution crime had reached 2672. It can be seen that the number of criminal cases of environmental pollution in China has generally increased in recent years.

Taking a province as an example, according to the statistics of the criminal judgments of the first instance of the crime of environmental pollution from 2015 to 2021, it can be seen that the number of cases of the crime of environmental pollution in a province has increased in multiples since 2015, but it can be seen that although the number of cases is still increasing every year since 2016, the growth rate shows a downward trend compared with previous years. This is because, in recent years, the problem of environmental pollution has become more and more serious, which has attracted the great attention of the government and relevant departments. The efforts to crack down on environmental pollution crimes have increased and achieved certain results. See Table 4.

### 4.2. Sample Data Analysis

From 2015 to 2018, due to the increased crackdown and supervision, the number of criminal judicial judgments on environmental pollution crimes also increased year by year, reaching a peak in 2015. After 2018, the environmental pollution of a province has been effectively controlled, the environmental protection situation has developed well, and the environmental protection policy has achieved certain results. See Figure 3.

The data change in Figure 3 fully shows that the judicial interpretation issued in the original legislative package has provided obvious help for the judicial organs to hear cases, which has rekindled the backlog of “trial passion.” In addition, the provincial party committee and the provincial government responded to the national call and put forward guidelines and measures for comprehensive environmental treatment, especially the supervision of water pollution, which also led to the surge in the number of cases. It can be seen that the increase in the number is the embodiment of the local government's attention to environmental protection [11–13].

The article "Reform and Analysis of the Division of Legal Responsibility between Enterprises and Third-Party Governance under Environmental Pollution" was published in 2022. Journal: J Environ Public Health.

As can be seen from Table 5, showing the basic situation of the application of freedom punishment in the cases of environmental pollution crime in a province from 2015 to 2021, after the establishment of the crime of environmental pollution, most of the penalties are concentrated in fixed-term imprisonment of less than 3 years, accounting for 60%; however, after 2018, it can be seen that among the number of people sentenced to freedom punishment, the number of suspended sentences has increased significantly, compared with the number of people sentenced to more than one year and less than three years [14]. See Figure 4.

In the 2099 cases, there were 815 cases of joint crime. Nearly 40% of the cases occurred in places where individuals illegally operated. Most environmental pollution cases were for the purpose of seeking benefits. Criminal acts need the cooperation of multiple people and division of labor; therefore, the majority of environmental pollution crimes are joint crimes. See Figure 5.

Among the 2099 judgments of first instance, there were 1894 natural person crimes, accounting for 90% of the total, 205 unit crimes, and accounting for 10% of the total, 12 people were exempted from criminal punishment. The number of people sentenced to probation, criminal detention, and fixed-term imprisonment of not more than three years was 3847, accounting for 97.6% of the total. Among them, 1393 were suspended, accounting for 35.3% of the total; 2093 people were sentenced to fixed-term imprisonment of less than three years, accounting for 53.1%. In comparison, the number of people exempted from punishment, single penalty, and fixed-term imprisonment of more than 3 years and less than 7 years is relatively small, of which 59 people are sentenced to fixed-term imprisonment of more than 3 years and less than 7 years, accounting for 1.5% of the total. 12 people were exempted from criminal punishment, accounting for 0.3% of the total. 23 people were fined only, accounting for 0.6% of the total. In judicial practice, the sentencing of most defendants of environmental pollution crime is relatively light (see Figure 6).

In terms of the types of criminal subjects, natural persons account for 90% of the subjects of environmental pollution crimes, and unit subjects account for only 10%. The subjects of environmental pollution crimes are mainly private workshops that conduct industrial processing and production privately or in violation of national regulations (see Figure 7).

As shown in Table 6, 80% of natural persons were fined less than 50000 yuan, accounting for 80.2% of the total number. Fines ranging from 50,000 yuan to 100,000 yuan accounted for 12.5% of the total number. In 2017, four defendants were fined more than 1 million yuan, and the highest was fined 3 million yuan. Among the accomplices, two defendants were fined 3 million yuan and one was fined 1.5 million yuan, which is a relatively high amount compared with other cases. However, generally speaking, the amount of fines for natural persons is relatively light [15–17].

The article "Reform and Analysis of the Division of Legal Responsibility between Enterprises and Third-Party Governance under Environmental Pollution" was published in 2022. Journal: J Environ Public Health.

As shown in Table 7, compared with natural person crimes, unit crimes account for only 10% of the total number of crimes, that is, 205 cases. However, in terms of the amount of fines, unit crimes are sentenced to more fines. 50 pieces less than 50,000 yuan; 71 pieces of RMB 50,000–150,000; 46 pieces of RMB 150,000–500,000; 11 pieces of RMB 500,000–1 million; 5 pieces of RMB 1–10 million; and for the two cases exceeding 10 million yuan, one was fined 18.5 million yuan and the other was fined 63 million yuan. There is a clear gap in the amount of fines for 17 unit crimes, most of which are concentrated below 500,000 yuan. Before 2019, most of the unit fines will be less than 150,000 yuan. After 2020, the penalty for units will increase [18, 19].

### 4.3. Cause Analysis

Of the total number of cases, the number of probation cases was up to 1049, accounting for about 49%. Probation cases are mostly concentrated in one year and six months a year, with a total of 713 cases. A total of 1393 people were sentenced to probation. The application of probation is different in the same province. At the same time, there is also uneven sentencing. Just like the three cases mentioned above, the pollution sources are generally the same or light, but the penalties are different. Some are applicable to probation, and some are not applicable [20]. See Table 8 for details.

As can be seen from Table 8, the first six items have legal commutation and discretionary commutation, and the last item can increase the sentence on the basis of the original sentence. These circumstances are the factors leading to the discretion of the judge. For the director of unit crime, if he is sentenced to fixed-term imprisonment, it may have a certain impact on the enterprise and local economy. The local government is under pressure to solve the employment problem of employees and the fluctuation of local finance. Under the influence of local protectionism, the government will intervene in the administration of justice, and the person in charge will also propose to pay more fines in exchange for the opportunity of probation [21–23].

## 5. Division of Responsibility for the Third-Party Treatment of Environmental Pollution of Enterprises

Due to the emergence of the third-party governance, the situation of single responsibility subject in the traditional model is broken, which makes the legal relationship of the third-party governance complex. The main characteristics are as follows: first, the diversification of responsibility subjects. In the traditional model, the subject of legal responsibility is only the sewage enterprises, while in the legal responsibility of third-party governance, the subject of responsibility includes sewage enterprises and environmental service companies [24]. Second, the sources of obligations of the subject of responsibility are different. The obligation of environmental service companies to treat the pollutants discharged by pollutant discharge enterprises comes from the contract between both parties and belongs to private law obligations. Third, the principle of responsibility has changed. Figures 8 and 9 show the legal relationship of environmental pollution control.

The article "Reform and Analysis of the Division of Legal Responsibility between Enterprises and Third-Party Governance under Environmental Pollution" was published in 2022. Journal: J Environ Public Health.

The third-party treatment contract of environmental pollution of the enterprise stipulates that the performance of the contract focuses on the pollution treatment process. The pollutant discharge enterprise fully trusts the environmental service company, and the payment of remuneration is not conditional on the third party achieving the expected effect of pollution treatment, then the rules of the entrustment contract can be applied to the contract. If the contract stipulates that the remuneration will be paid only when a certain governance effect is achieved, the rules of contract for work shall apply.

### 5.1. Division of Civil Liability

The division of civil liability can implement the governance mode of entrusting a third party to operate.

In the entrusted governance model, pollutant discharge enterprises have ownership and control over pollution production equipment, pollution control equipment, and pollutants. According to whether there is fault between the pollutant discharge enterprise and the environmental service company, it can be divided into the following five situations:

First, the pollutant discharge enterprise and the environmental service company have common faults, which constitute joint infringement. It is generally believed that joint tort can include joint negligence, not limited to joint intention. As joint infringement produces joint and several liability, both parties shall bear joint and several liability for compensation.

Second, both sewage enterprises and environmental service companies have faults for environmental infringement, but they do not belong to common faults. Since the pollutant discharge enterprises have the ownership and control over the pollution production equipment and pollution control equipment, and the pollutant discharge enterprises are responsible for the pollution discharge behavior, the pollutant discharge enterprises shall bear the environmental tort liability alone. However, bearing the tort liability does not affect the investigation of the liability for breach of contract. After assuming the tort liability, the pollutant discharge enterprise can recover the damage caused by the breach of contract of the environmental service company.

The article "Reform and Analysis of the Division of Legal Responsibility between Enterprises and Third-Party Governance under Environmental Pollution" was published in 2022. Journal: J Environ Public Health.

Third, the sewage enterprises and environmental service companies are not at fault. Because the principle of no fault liability is applicable to environmental tort, regardless of the perpetrator's illegality and subjective fault, up to standard discharge and no fault cannot become the exemption cause of environmental pollution liability, and the polluter still has to bear tort liability. In other words, when the pollutant discharge enterprises and environmental service companies fulfill their respective obligations according to the contract and achieve up to standard discharge, but still cause environmental pollution damage, the polluter shall still bear the responsibility. Since the pollutant discharge enterprise has the ownership and control over the pollution production equipment and pollution control equipment, and has implemented the pollutant discharge behavior, the polluter should be the pollutant discharge enterprise, and the pollutant discharge enterprise should bear the tort liability [25].

Fourth, the pollutant discharge enterprise is at fault, and the environmental service company is not at fault. The environmental service company provides treatment services according to the contract, but the pollutant discharge enterprise does not discharge the type, concentration, and quantity of pollutants according to the contract, resulting in damage. At this time, there is a causal relationship between the behavior of the pollutant discharge enterprise and the damage results, and the pollutant discharge enterprise has the ownership and control over the pollution production equipment and pollution control equipment, so the pollutant discharge enterprise should bear the environmental tort liability.

Fifth, the pollutant discharge enterprises are not at fault, and the environmental service companies are at fault; for example, the pollutant discharge enterprises discharge pollutants according to the types, concentrations, and quantities of pollutants agreed in the contract, but the environmental service companies do not operate the pollution control equipment normally in the process of pollution control and illegally discharge pollutants, resulting in damage consequences. Since the pollutant discharge enterprises have the ownership and control over the pollution production equipment and pollution control equipment, and learn from the environmental equipment liability theory, the pollutant discharge enterprises shall bear the environmental tort liability. After assuming the tort liability, the pollutant discharge enterprise has the right to request the environmental service company to bear the corresponding liability for breach of contract in accordance with the environmental service contract signed by both parties.

The article "Reform and Analysis of the Division of Legal Responsibility between Enterprises and Third-Party Governance under Environmental Pollution" was published in 2022. Journal: J Environ Public Health.

### 5.2. Division of Administrative Responsibility

#### 5.2.1. Division of Responsibilities in Entrusted Operation Third-Party Governance

In the commissioned third-party treatment, as the manufacturer of pollution sources, the pollutant discharge enterprise must be the supervision object of the competent administrative department, and the pollutant discharge enterprise has the ownership and control over the pollution treatment equipment and pollutants. Therefore, even for the reasons of environmental service companies, the pollutant discharge enterprise should also bear administrative responsibility. For the environmental service company, it mainly sends technicians to settle in the sewage discharge enterprise, manage the sewage treatment equipment, and treat the pollutants. Therefore, the environmental service company does not have external independence and will not bear administrative responsibility in case of illegal sewage discharge. However, if the illegal sewage discharge is caused by the environmental service company's laziness in governance or illegal breach of contract, the sewage discharge enterprise can recover from it after taking responsibility as a “polluter.”

#### 5.2.2. Division of Responsibilities in Building Operational Third-Party Governance

In the construction and operation of third-party governance, pollutant discharge enterprises are still the manufacturers of pollution sources, which is obviously the supervision object of the competent environmental administrative department. Since environmental service companies enjoy pollution control equipment and have the right to control and dominate pollutants, and they are also the main body that ultimately discharges pollutants to nature, they can be included in the scope of “enterprises and institutions discharging pollutants” stipulated by law by expanding the interpretation of “polluters” and become the supervision object of the competent environmental administrative department. The division of administrative responsibility for the construction of operational third-party governance needs to divide the responsibilities of both parties according to the main reasons that lead to the failure to complete the governance task.

The article "Reform and Analysis of the Division of Legal Responsibility between Enterprises and Third-Party Governance under Environmental Pollution" was published in 2022. Journal: J Environ Public Health.

First, if the pollution discharge enterprise and the environmental service company are caused by common reasons, both parties shall bear corresponding administrative responsibilities. Common reasons include illegal discharge of pollutants after negotiation by both parties or similar situations such as excessive discharge of pollutants caused by the operation failure of pollution control equipment when the environmental service company is treating pollutants due to the failure of pollutant treatment equipment. At this time, the competent department of ecological environment shall punish both parties in accordance with the environmental administrative laws and regulations.

Second, only for the reasons of pollutant discharge enterprises, the polluters should bear the administrative and legal responsibility for illegal pollutant discharge; for example, the environmental service company cannot complete the treatment task because the pollutant discharge enterprise does not discharge the type and quantity of pollutants according to the contract. The reasons are as follows: first, whether independent or embedded, both sides can implement pollution discharge behavior relatively independently; and second, the premise for the transfer of pollution control responsibility of pollutant discharge enterprises is that their own production and operation behavior is legal, and the quantity, concentration, and other indicators of pollutants delivered to environmental service companies comply with legal provisions and contract agreements. Therefore, at this time, pollutant discharge enterprises should bear the administrative and legal responsibility for illegal pollutant discharge and bear the corresponding liability for breach of contract to environmental service companies.

Third, only for the reason of environmental service company, the environmental service company shall bear the administrative responsibility. The pollutant discharge enterprise carefully selects a qualified environmental service company and discharges pollutants according to the contract. However, if the environmental service company fails to complete the treatment task due to the fault of the pollution treatment equipment or staff of the environmental service company, the environmental service company shall bear the corresponding administrative responsibility; if the environmental service company breaches the contract to the pollutant discharge enterprise, it shall bear the corresponding liability for breach of contract at the same time. The government should speed up the construction of the credit rating system of environmental service companies, which is conducive to judging whether the pollutant discharge enterprises have fulfilled their duty of prudence.

The article "Reform and Analysis of the Division of Legal Responsibility between Enterprises and Third-Party Governance under Environmental Pollution" was published in 2022. Journal: J Environ Public Health.

### 5.3. Division of Criminal Responsibility

For the environmental criminal responsibility of the third-party treatment of environmental pollution of enterprises, this paper will no longer distinguish between the entrusted operation mode and the construction operation mode. Because the ownership and control of pollutants and their production equipment do not affect the establishment of the crime of environmental pollution, the identification of the criminal responsibility of sewage enterprises and third parties depends on whether they meet the constitutive elements of the crime of environmental pollution. However, the subjective elements of the crime of polluting the environment are still controversial. The author believes that the principle of legality should be strictly followed, and negligence cannot constitute the crime of polluting the environment. For the negligent discharge of pollutants by pollutant discharge enterprises or environmental service companies, which has caused serious consequences, civil compensation and administrative punishment cannot achieve the purpose of punishment. Illegal pollutant discharge substances can be identified as toxic substances in dangerous substances, and criminals can be punished through the crime of negligent release of dangerous substances.

In the third-party governance model of enterprise environmental pollution, the subjects constituting the crime of environmental pollution include sewage enterprises and their supervisors, directly responsible personnel, environmental service companies and their supervisors and directly responsible personnel. Since the number of people involved may be large, the principle of legality must be strictly observed to ensure fairness and justice. Neutral duty behavior can be the obstruction of the objective elements of the crime. However, as long as the behavior is not implemented by following the arrangement of the leader, it is a neutral job behavior, which should be analyzed in combination with its own work content. In addition, it is worth mentioning that in order to encourage the subject of responsibility to repair the ecological environment, the law stipulates that the active implementation of civil compensation and administrative fines will be conducive to the sentencing of the crime of environmental pollution. The starting point of this provision is good, but we should be careful that “replacing punishment with punishment” will affect judicial fairness.

In the third-party treatment mode of enterprise environmental pollution, if both parties jointly deliberately commit the criminal act, the pollutant discharge enterprise and its supervisors, the persons directly responsible and the environmental service company and its supervisors, and persons directly responsible shall be recognized as joint crimes, the pollutant discharge enterprise and the environmental service company shall be fined, and their supervisors and persons directly responsible shall be punished in accordance with the provisions of natural persons committing the crime. If one party of a pollutant discharge enterprise or environmental service company knows the other party's criminal act and still provides convenience for the other party, it can be identified as a one-sided accomplice and punished according to the former situation. If there is no evidence to prove that the pollutant discharge enterprise and the environmental service company constitute joint intention, if the environmental service company has committed the criminal act, the environmental service company and its supervisors and directly responsible personnel shall bear criminal responsibility; and if the environmental service company is not aware of the criminal act committed by the pollutant discharge enterprise, the pollutant discharge enterprise and its supervisors and directly responsible personnel shall bear criminal responsibility.

The article "Reform and Analysis of the Division of Legal Responsibility between Enterprises and Third-Party Governance under Environmental Pollution" was published in 2022. Journal: J Environ Public Health.

## 6. Conclusion

Since the crime of environmental pollution is a double punishment system, the unit can also constitute the crime. According to the statistical table of unit crime, out of a total of 2099 judgments, there are only 205 cases involving unit crime, accounting for 10% of the total, and the remaining natural person crimes account for 90%. The units of environmental pollution administrative punishment cases account for a large proportion, reaching about 91%. Through the research, it is found that an important condition for the establishment of unit crime is that the criminal act must reflect the will of the unit. However, the definition of unit will is vague, and there is no explicit legislation, but this identification is handed over to the theoretical and practical circles. In this case, the court held that the defendant illegally discharged sewage according to his personal will and did not reflect the will of the unit. Only one defendant was sentenced to fixed-term imprisonment, and the other two defendants were sentenced to probation. It is generally believed that the first consideration is whether the pollution discharge behavior has undergone the collective research and decision-making of the unit or the decision of the person directly in charge because if the behavior is not the case, it must not be a unit crime. But sometimes superficial does not necessarily reflect the will of the unit. In the process of performing tasks, employees may often hand over hazardous wastes to enterprises without waste treatment qualification to improve efficiency and profits, but it is uncertain whether this is the will of the unit; whether it can also be recognized as the interests of the unit that senior executives use the unit's vehicles to help their friends deal with hazardous waste for the sake of human relations is controversial.

The article "Reform and Analysis of the Division of Legal Responsibility between Enterprises and Third-Party Governance under Environmental Pollution" was published in 2022. Journal: J Environ Public Health.

However, the development of the third-party governance model of enterprise environmental pollution has injected vitality into the industrial market, enabling enterprises to control pollutants efficiently and at low cost and narrowing the governance responsibility and supervision scope of the government. Therefore, the central and local governments have vigorously promoted the third-party governance model of environmental pollution. However, due to the novelty of this model, there is no systematic provision in China's existing legal system, resulting in a cluster of problems in judicial practice. Therefore, we must further clarify the division of legal liability for environmental pollution. In addition to studying the legal liability of third-party governance of environmental pollution of enterprises, how to reduce the risk of loss caused by environmental pollution and reduce the cost of pollution governance is another issue worthy of discussion.

The environmental service market can further explore the construction of environmental liability insurance system and the establishment of damage compensation foundation for environmental service enterprises, so as to improve the anti-risk ability of pollutant discharge enterprises and environmental service companies. If we want to promote the third-party governance model, we should firmly grasp the current policy opportunities and be based on the actual needs. At the national level, while supporting the third-party governance system of environmental pollution, we also need to actively explore the internal management methods of the system; for example, formulate project bidding and acceptance standards to promote the third-party governance system to be more mature and standardized. In addition, we should also introduce more detailed and practical legal regulations as soon as possible to facilitate the implementation of the third-party governance system.

## Figures and Tables

**Figure 1:** Problems faced by enterprises and third-party governance under environmental pollution.

**Figure 2:** Statistics on the number of environmental pollution crime cases concluded by courts at all levels in the first instance from 2015 to 2021.

The article "Reform and Analysis of the Division of Legal Responsibility between Enterprises and Third-Party Governance under Environmental Pollution" was published in 2022. Journal: J Environ Public Health.

**Figure 3:** Number of environmental pollution crime cases concluded by courts at all levels of a province in the first instance from 2015 to 2021.

**Figure 4:** Joint crime and non-joint crime of environmental pollution crime concluded by courts at all levels of a province in the first instance from 2015 to 2021.

**Figure 5:** Punishment of environmental pollution crime concluded by courts at all levels of a province in the first instance from 2015 to 2021.

**Figure 6:** Number of crimes committed by environmental pollution crime units concluded by courts at all levels of a province in the first instance from 2015 to 2021.

**Figure 7:** Subjects of environmental pollution crimes concluded by courts at all levels of a province in the first instance from 2015 to 2021.

**Figure 8:** Legal relationship of traditional environmental pollution control.

**Figure 9:** Legal relationship of third-party treatment of environmental pollution of enterprises.

**Table 1:** Comparison between “major pollution crime” and “environmental pollution crime.”

	Charge	Range of pollutants	Lower threshold of conviction	Object expansion	Immediate standard
97 Criminal Law	Crime of major environmental pollution accident	“Radioactive other hazardous waste”	“Causing major environmental pollution, casualties, and serious consequences”	“Disposal to land and water”	“Major property losses or personal casualties”
Criminal Law Amendment VIII	Crime of environmental pollution	Replace “other hazardous wastes” with “other hazardous substances”	“Seriously polluting the environment”	Cancel the list of objects and replace it with “violation of national regulations”	Serious environmental pollution

**Table 2:** Comparison of environmental pollution crime and penalty between “Criminal Law Amendment 8” and “Criminal Law Amendment 11.”

	Legal punishment grade	Maximum sentence	Determination of the circumstances of “fixed-term imprisonment of not less than three years but not more than seven years”	When competing with other crimes
Criminal Law Amendment VIII	Grade 2 “serious environmental pollution” and “especially serious consequences”	If the consequences are especially serious, he shall be sentenced to fixed-term imprisonment of up to seven years	The consequences are particularly serious	Nothing

Criminal Law Amendment 11	Grade 3 “serious environmental pollution,” “serious circumstances,” “four felony cases applicable to a prison term of more than seven years”	Under any of the following four circumstances, the maximum term of imprisonment is 15 years	Serious circumstances	Be convicted and punished in accordance with the provisions on heavier punishment

The article "Reform and Analysis of the Division of Legal Responsibility between Enterprises and Third-Party Governance under Environmental Pollution" was published in 2022. Journal: J Environ Public Health.

**Table 3:** Sample data of environmental pollution crime cases from 2015 to 2021.

Grassroots court		Intermediate court	High court	
12,699		3389	30	

*Trial procedure*				
First instance	Second instance	Trial supervision	Penalty and execution change	Other
12,754	2458	114	814	4

*Text type*				
Judgment	Ruling	Conciliation statement	Decision	Notice
12,778	3187	7	81	88

**Table 4:** Number of first instance cases of “environmental pollution crime” in a province from 2015 to 2021.

Particular year	2015	2016	2017	2018	2019	2020	2021
	20	461	506	414	245	201	188

**Table 5:** Number of natural persons punished for environmental pollution crimes concluded by courts at all levels of a province in the first instance from 2015 to 2021.

Particular year	Exemption from punishment	Single penalty	Probation	Criminal detention	3–7 years	Total
2015	0	0	3	17	2	22
2016	0	3	172	502	20	697
2017	2	1	251	501	8	763
2018	3	5	322	376	1	707
2019	4	5	184	176	7	385
2020	0	3	178	143	16	340
2021	0	1	217	131	20	369

**Table 6:** Number of natural person fines for environmental pollution crimes concluded by courts at all levels of a province in the first instance from 2015 to 2021.

Particular year	Less than 5	5–10	10–20	20–50	50–100	More than 100
2015	22	3	0	0	0	0
2016	736	30	32	3	0	0
2017	727	134	57	5	1	4
2018	626	90	53	8	0	0
2019	374	47	4	4	1	0
2020	312	45	32	6	0	0
2021	271	76	33	6	2	0

**Table 7:** Fines of environmental pollution crime units concluded by courts at all levels of a province in the first instance from 2015 to 2021.

Particular year	Less than 5	5–15	15–50	50–100	100–1000	More than 1000
2015	0	0	0	0	0	0
2016	9	12	2	1	0	1
2017	4	13	11	1	2	1
2018	16	20	4	3	1	0
2019	12	7	3	1	1	0
2020	6	9	12	2	0	0
2021	3	10	14	5	1	0

**Table 8:** Application of sentencing circumstances of environmental pollution crime concluded by courts at all levels of a province in the first instance from 2015 to 2021.

	Sentencing circumstances	Number of cases	Case number
1	Confess	153	(2013) Jin Pu criminal procedure of first instance No. 765, etc
2	Render meritorious service	64	(2014) Jin Pu criminal procedure of first instance No. 187, etc
3	Surrender oneself	604	(2014) Yu Yu criminal procedure of first instance No. 151, etc
4	Accessory	369	(2015) Wen Le criminal procedure of first instance No. 1573, etc
5	First offense, incidental offense	99	(2015) Tai Lu criminal procedure of first instance No. 271, etc
6	Pay environmental remediation fee	35	(2019) Zhe 0602 criminal procedure of first instance No. 1172, etc
7	Recidivism	26	(2015) Wen Le criminal procedure of first instance No. 959, etc

## Data Availability

The labeled data sets used to support the findings of this study are available from the corresponding author upon request.

The article "Reform and Analysis of the Division of Legal Responsibility between Enterprises and Third-Party Governance under Environmental Pollution" was published in 2022. Journal: J Environ Public Health.

## References

[1] Austin A. (2019). Arborist reporting standards legal liability for the consultinq arborist. *Environmental and Planning Law Journal*.

[2] Kuzmin I. A. (2019). Problems and prospects of improving the legal construction of legal liability in the field of investment legal relations. *Juridical Journal of Samara University*.

[3] Kozhevnikov V. V. (2021). On functional purpose of legal liability. *SIASAT*.

[4] Zamroni M. (2020). Legal liability of advocates in legal services contracts. *Substantive Justice International Journal of Law*.

[5] Bakumov O. S. (2019). Ensuring the state’s legal liability is the key challenge of legal reform in the modern Ukraine. *Bulletin of Kharkiv National University of Internal Affairs*.

[6] Alimova A. I. (2020). Problems of legal liability of the employer (according to article 145.1 of the criminal code of the Russian federation). *Bulletin of Udmurt University. Series Economics and Law*.

[7] Gea A. F., Hirsanuddin H., Djumardin D. (2020). Tanggung jawab direksi atas terjadinya pailit perseroan terbatas. *JESS (Journal of Education on Social Science)*.

[8] Guan Y., Zhang L., Zheng L., Zou H. (2021). Managerial liability and corporate innovation: evidence from a legal shock. *Journal of Corporate Finance*.

[9] Ernst J., Mansberger R., Muggenhuber G., Navratil G., Twaroch C. (2019). The legal boundary cadastre in Austria: a success story?. *Geodetski Vestnik*.

[10] Martono D. B., Aditya T., Subaryono S., Nugroho P. (2021). The legal element of fixing the boundary for Indonesian complete cadastre. *Land*.

[11] Asmuni A., Kurniawan K., Bayo E. (2019). Liabilities of the director of the regional limited liability company (perseroda) in the corporate bankruptcy according to positive law. *International Journal of Multicultural and Multireligious Understanding*.

[12] Taveriyanto A., Andiyarto H. T. C., Saefullah M. V., Haliza M. P. (2022). The utilization of gypsum board and fly ash waste on brick in terms of compressive strength to reduce environmental pollution. *IOP Conference Series: Earth and Environmental Science*.

[13] Wang L. (2022). Role of fdi and energy intensity in mitigating the environmental pollution in the Chinese steel industry: does technological innovation makes a difference?. *Environmental Science and Pollution Research*.

[14] Cazzolla Gatti R. (2021). Why we will continue to lose our battle with cancers if we do not stop their triggers from environmental pollution. *International Journal of Environmental Research and Public Health*.

[15] Sun F., Benn M., Bernhardt K., Li W.-H., Liu-Walsh F., Yang A. Y. (2021). 27027 mitigation of damage induced by environmental pollution by feverfew extract. *Journal of the American Academy of Dermatology*.

The article "Reform and Analysis of the Division of Legal Responsibility between Enterprises and Third-Party Governance under Environmental Pollution" was published in 2022. Journal: J Environ Public Health.

[16] Mondol M., Sani A., Usha K., Marzia S., Biswash P., Islam M. (2021). Exploring rice residue management practices focusing environmental pollution and soil health in six major rice growing upazilas of mymensingh district in Bangladesh. *Progressive Agriculture*.

[17] Cygańczuk K., Janik P. (2021). The threat of environmental pollution with harmful substances, on the example of uncontrolled fires in landfills and actions aimed at reducing it. *Safety & Fire Technology*.

[18] Pawowski W., Karpińska M. (2021). The effect of soil moisture on the ability to detect tnt pairs from the sand layer in order to prevent environmental pollution and groundwater. *Molecules*.

[19] Astaneh N., Bazrafshan F., Zare M., Amiri B., Bahrani A. (2021). Nano-fertilizer prevents environmental pollution and improves physiological traits of wheat grown under drought stress conditions. *Scientia Agropecuaria*.

[20] Sari D. K., Waremra R. S., Setiawan M. R. E. (2021). The energy change props from used goods to reduce impact of environmental pollution in the land of anim ha. *IOP Conference Series: Materials Science and Engineering*.

[21] Montecchi M., Plangger K., West D. C. (2021). Supply chain transparency: a bibliometric review and research agenda. *International Journal of Production Economics*.

[22] Salza P., Palomba F., Di Nucci D., De Lucia A., Ferrucci F. (2020). Third-party libraries in mobile apps. *Empirical Software Engineering*.

[23] Lin Y.-D., Truong D.-T., Ali A., Li C.-Y., Lai Y.-C., Dinh T.-M. T. (2020). Proxy-based federated authentication: a transparent third-party solution for cloud-edge federation. *IEEE Network*.

[24] Aureliu-Florin H., Popa B., Heras-Saizarbitoria I., Boiral O., Abrudan I. V. (2021). Procedural factors influencing forest certification audits: an empirical study in Romania. *Forests*.

[25] Ulutaş A., Topal A. (2022). A new hybrid model based on rough step-wise weight assessment ratio analysis for third-party logistics selection. *Soft Computing*.

